# Resveratrol Inhibits Invasion and Metastasis of Colorectal Cancer Cells via MALAT1 Mediated Wnt/β-Catenin Signal Pathway

This article has been retracted.

**DOI:** 10.1371/journal.pone.0078700

**Published:** 2013-11-11

**Authors:** Qing Ji, Xuan Liu, Xiaoling Fu, Long Zhang, Hua Sui, Lihong Zhou, Jian Sun, Jianfeng Cai, Jianmin Qin, Jianlin Ren, Qi Li

**Affiliations:** 1 Department of Medical Oncology, Shuguang Hospital; Shanghai University of Traditional Chinese Medicine, Shanghai, China; 2 Interventional Cancer Institute & Department of General Surgery, Shanghai University of Traditional Chinese Medicine, Shanghai, China; 3 Department of Chemistry, University of South Florida, Tampa, Florida, United States of America; 4 Department of Oncology, Shanghai Municipal Hospital of Traditional Chinese Medicine, *S*hanghai, China; Florida International University, United States of America

## Abstract

Resveratrol, extracted from Chinese herbal medicine Polygonum cuspidatum, is known to inhibit invasion and metastasis of human colorectal cancer (CRC), in which long non-coding Metastasis Associated Lung Adenocarcinoma Transcript 1 (RNA-MALAT1) also plays an important role. Using MALAT1 lentiviral shRNA and over-expression constructs in CRC derived cell lines, LoVo and HCT116, we demonstrated that the anti-tumor effects of resveratrol on CRC are through inhibiting Wnt/β-catenin signaling, thus the expression of its target genes such as c-Myc, MMP-7, as well as the expression of MALAT1. In detail, resveratrol down-regulates MALAT1, resulting in decreased nuclear localization of β-catenin thus attenuated Wnt/β-catenin signaling, which leads to the inhibition of CRC invasion and metastasis. This finding of ours surely provides important pre-clinical evidence supporting future use of resveratrol in prevention and treatment of CRC.

## Introduction

Colorectal cancer is the results of the mutation of multiple genes including proto-oncogenes and tumor suppressor genes. As the oncogenes controlling cell proliferation remaining highly expressed, or the tumor suppressor genes being mutated, the resulting cancerous cells evade immune system, form tumors in distal locations/organs, i.e. metastasis and the terminal stage of cancer begins [1].

The emergence of new Chinese medicine monomer anticancer drugs has provided a new option to the reptoire of synthetic drugs for cancer treatment [2]. Polygonum cuspidatum is the rhizomes and root of the Tateshina perennial herb - Polygonum cuspidatum [3]. Previous data showed that Polygonum cuspidatum had various inhibitory effects on tumor, bacterial/viral infections and inflammation [3]–[7]. Resveratrol extracted from Polygonum cuspidatum is a natural antioxidant, which can reduce blood viscosity, inhibit platelet aggregation and vasodilation, maintain the blood flow, and prevent the occurrence and development of cancer [8]–[10].

Early in 2003, Ji *et al* firstly identified long non-coding RNA - MALAT1. In 225 cases of stage I non-small cell lung cancer (NSCLC), it was found in 70 cases, metastasis correlates with MALAT1 over-expression, in a course and tissue specific manner, suggesting that MALAT1 expression can serve as a potential marker of survival in stage 1 NSCLC patients [11]. Furthermore, other groups showed that MALAT1 over-expresses in liver, cervical and colon cancer [12]–[14].

Many studies have shown that Wnt/β-catenin signaling pathway regulates tumor cell invasion and metastasis. Soichi *et al* found that in oral squamous cell carcinoma cells, the accumulation of β-catenin in the cytoplasm induces TCF/LEF transcriptional activity, and increase the MMP-7 expression, thereby inducing the conversion of epithelial cells to mesenchymal cells as well as enhancing invasion and metastasis [15]. Guo *et al* demonstrated in CRC HT29 cell line, NGX6 gene product inhibited transferring of the β-catenin from the nucleus and cytoplasm to the cell membrane, thereby inhibiting the transcriptional activity of TCF and down-regulating the expression of Wnt target genes c-Myc, cyclinD1 and COX-2, leading to decreased cancer cell invasion and metastasis [16].

Our present studies interrogated the mechanisms by which resveratrol regulates MALAT1 and Wnt/β-catenin signal pathway, resulting in repressed cancer cell invasion and metastasis.

## Materials and Methods

### In Situ Hybridization on Tissue Samples from Patients with CRC

Paraffin-embedded tumor and adjacent normal tissue samples from 60 CRC patients who underwent tumor resection at Putuo Hospital, Shanghai University of Traditional Chinese Medicine (SUTCM)between 2010 and 2012 were selected for hybridization with digoxigenin (DIG)-labeled MALAT1 DNA probe (Shinegene Molecular Biotechnology, Shanghai, China). The experiment was performed according to the method described by Tanner *et al* [17]. The study was approved by the ethic committee of Pu Tuo Hospital, SUTCM and all patients were provided with written informed consent.

### Screening of Chinese Medicine Monomer Anticancer Drugs on MALAT1 Expression in LoVo Cells

LoVo cells (derived from left supraclavicular region metastasis, Dukes’ type C, grade IV, colorectal adenocarcinoma) were cultured in F12K medium supplemented with 10% fetal bovine serum, 100 g/ml streptomycin, 100 U/ml penicillin, at 37°C, 5% CO2, and high humidity. All the Chinese medicine monomer anticancer drugs were diluted serially to detect the half inhibition concentration on proliferation of LoVo cells. Proliferation of LoVo cells was determined by Cell Counting Kit-8 (CCK-8) assay as described previously [18]. Real time PCR was used for detecting the inhibition rate of candidate drugs on MALAT1 expression. For real time PCR analysis, the forward primer, the reverse primer, and the Taqman probe were designed as follows: forward (5-AGGCGTTGTGCGTAGAGGA-3), reverse (5-GGATTTTTACCAACCACTCGC-3), TaqMan probe (5-fam+CCTAGACCAGCATGCCAGTGTGCC+tamara-3). Real time PCR was performed in the Applied Biosystems 7300 System (Applied Biosystems Deutschland GmbH) using Premix Ex Taq (Takara, DaLian, China). GAPDH was used as internal reference.

### Knockdown and Over-expression of MALAT1 Gene

Human MALAT1 cDNA (Gene ID: 378938) was amplified by RT-PCR with the RNA extracted from LoVo cells, and then cloned into pLV4 vector. MALAT1 were searched for suitable siRNA target sequences, three siRNA sequences were designed, synthesized, and confirmed by sequencing respectively. Lentiviral particles were produced by co-transfecting expression vector pLV4-MALAT1 cDNA or pLV4-MALAT1 shRNA with viral particle packaging helper vector into 293T cells. Preliminary experiments picked out the most efficient siRNA sequences of knockdown from the above mentioned three candidate siRNA (Figure S1): sense 5′-GAGGUGUAAAGGGAUUUAUTT-3′, anti-sense 5′-AUAAAUCCCUUUACACCUCTT-3′; with a negative control siRNA sequence: sense 5′-UUCUCCGAACGUGUCACGUTT-3′, anti-sense 5′-ACGUGACACGUUCG.

GAGAATT-3′. Titer of viral particles containing MALAT1 shRNA and MALAT1 cDNA was determined by limited serial dilution. The efficiency of knockdown or over-expression was determined by real time PCR. LoVo cells or HCT116 cells were infected with the lentivirus with the pLV4-MALAT1 cDNA, pLV4-MALAT1 shRNA or pLV4-vector.

### Luciferase Reporter Assay

To test MALAT1 promoter or LEF/TCF promoter activity, LoVo cells were co-transfected with either the recombinant plasmid pGL3-basic-MALAT1 promoter or pGL3-basic-LEF/TCF promoter with a control positive plasmid pRL-SV40 as previously described [19]. The promoter activity was analyzed using a commercial dual-luciferase assay kit (Beyotime Institute of Biotechnology, China) according to the manufacturer’s instructions.

### Migration and Invasion Assay

A total of 5×10^5^ LoVo cells cultured in 100 µl F12K with 0.5% FBS were seeded into the upper part of a transwell chamber (Corning Incorporated, Corning, NY). For migration analysis, in the lower part of the chamber, 600 µl F12K with 15% FBS and 10µg/ml fibronectin was added and the assay was performed for 24 hours at 37°C and 5% CO2. Migrated cells were analyzed by crystal violet staining, followed by observing under a DMI3000 B inverted microscope (Leica, Germany). For invasion analysis, 100 µl matrigel (BD, USA) was firstly added unto the bottom of the transwell chamber before LoVo cells were seeded, and the following procedures were the same as migration analysis, except for the invasive cells being analyzed after co-culture for 48 hours. As to HCT116 cells, the procedures were similar, the only difference was cells being cultured with RIPM 1640.

### Western Blot

Whole cell, cytoplasm, and nuclear proteins from LoVo or HCT116 cells were prepared according to the manufacturer’s instructions of ProteoJET Cytoplasmic and Nuclear Protein Extraction Kit (Fermentas, USA). Proteins were loaded onto the SDS-PAGE gels for electrophoresis, transferred to PVDF membranes and blocked in 5% milk prior to incubation with the indicated primary antibodies and the secondary antibodies. The resulting immunocomplexes were visualized by enhanced chemiluminescence. Protein loading was normalized by β-actin (whole protein or cytoplasm protein) or PCNA (nuclear protein).

### RNA-binding Protein Immunoprecipitation

RNA-binding protein immunoprecipitation (RIP) was performed according to the manufacturer’s protocols from the EZ-Magna RIP Kit (Millipore, USA). Briefly, LoVo cells were rinsed with ice-cold phosphate buffered saline (PBS), lysed by RIP lysis buffer. Both β-catenin (CST, USA) and nonspecific control rabbit IgG antibodies were used for the immunoprecipitation. RIP lysates and magnetic beads-bound β-catenin antibody were incubated together with rotating for overnight at 4°C. Afterwards, proteins in the immunoprecipitate were digested with proteinase K and bound RNAs were purified from the supernatants, reverse-transcribed using PrimeScript RT reagent Kit followed by quantitative analysis.

### Inmunofluorescence Microscopy

LoVo cells (2.5×10^5^) were grown on chamber slides (Millipore, USA) for 8 hours, starved for 12 hours. Cells were fixed for 40 minutes with 4% paraformaldehyde in PBS at room temperature, permealized and blocked with 5% non-fat dry milk, 1% BSA, 0.5% Triton X-100 and incubated overnight with rabbit monoclonal anti-β-catenin (CST, USA). After washing the slides, Cy3-conjugated anti-rabbit IgG antibody (Beyotime Institute of Biotechnology, China) was added in blocking solution for 1 hour. 4–6-diamidino-2-phenylindole was applied to stain nuclei. Immunofluorescence images were taken with a DMI3000B inverted microscope (Leica, Germany).

### Statistical Analysis

All data were presented as means SEM. The mean values of two groups were compared by Student’s *t* test. The associations between the expression of MALAT1 and clinicopathological parameters were analyzed using Fisher’s exact test, chi-square tests or continuity correction chi-square tests by SPSS18.0 software.

## Results

### 1. MALAT1 is Overexpressed in the Colorectal Cancer Tissues and Correlates with Tumor Metastasis and Invasion

Using *in situ* hybridization, we found there was higher expression of MALAT1 in the colorectal cancer tissue (CRC) than the adjacent normal colorectal tissue (Figure 1 and Table 1). We next conducted correlation analysis between MALAT1 expression and clinicopathological characteristics of CRC. A statistically significant association was observed between MALAT1 expression and extent of metastasis and invasion. In contrast to adjacent normal tissues, the MALAT1 expression in CRC tissues resected from patients with metastatic diseases was higher than those with no metastasis (Table 2). This association between MALAT1 expression and extent of metastasis and invasion was also confirmed by real time PCR (Figure S1).

**Figure 1:** Overexpression of MALAT1 in human colorectal cancer tissues. *In situ* hybridization was applied to investigate the MALAT1 expression in 60 paraffin-embedded tumor tissue and adjacent normal tissue samples of CRC patients.

**Table 1:** In situ hybridization of MALAT1 in human CRC tissues.

Tissues	Case	Staining intensity						*p* value
			–	+/−	+	++	+++	
tumors*	60		3	4	19	25	9	0.000
adjacentnormal	60		36	13	11	0	0	

* : *p*<0.01 vs. adjacent normal tissues.

**Table 2:** MALAT1 overexpression correlates with invasion and metastasis of human CRCs.

Variable	Cases		MALAT1expression							*p* value	
			negative		positive						
**Gender**											
Male		25		3		3			0.205		
Female		35		22		20					
**Age**											
<60		31		4		4		0.268			
≥60		29		31		33					
**Tumor size(** ***d/*** **cm)**											
*d*<6		41		4		1	0.446				
*d*≥6		19		27		38					
**Degree of differentiation**											
Poorly		23		3		6	0.334				
Moderately and well		37		26		15					
**Extent of invasion and metastasis**											
Yes		39		5		4	0.031*				
No		21		36		32					
**Duke’s stage**											
A–B		36		2		3	0.254				
C–D		24		17		21					

* : *p*<0.05 vs. no invasion and metastasis group.

### 2. Resveratrol Inhibits Proliferation, Migration and Invasion of LoVo Cells

To screen Chinese medicine monomer anticancer drugs which inhibited MALAT1 expression in LoVo cells, we first investigated the impact of candidate drugs on the proliferation of LoVo cells, and calculated the half inhibition concentration (IC50) of all candidate drugs (Table 3). Next we looked into the effect of candidate drugs on the inhibition of the MALAT1 expression. Our results demonstrated that resveratrol and osthole were the 2 top anticancer drugs with regard to inhibiting MALAT1 expression, with the resveratrol being the best one among these two (Figure 2A). Therefore, we chose resveratrol for our further studies on MALAT1 and related mechanisms. With our data showing an resveratrol IC50 of 55 µM in the LoVo cells (Figure 2B), the drug doses of 15, 30 and 50 µM were thus chosen for investigating of resveratrol’s effect on the invasion and migration capabilities of the cancer cells. Our results showed LoVo cells were significantly inhibited on their ability to invade and migrate by resveratrol, in a dose-dependent manner (Figure 2C).

**Figure 2:** Resveratrol inhibites the proliferation, migration and invasion of CRC LoVo cells. (A): Twenty-two candidate Chinese medicine monomer anticancer drugs were tested for the effective inhibition doses on the MALAT1 expression in LoVo cells. (B): Correlation of resveratrol drug doses and growth inhibition in LoVo cells. Y axis: percentage of growth inhibition; X axis: resveratrol concentrations (µM). (C): Assessment and quantification of cell migration and invasion of LoVo cells. Values represent the number of migratory/invasive cells per 5 high power fields. *p<0.05 or **p<0.01, compared with control LoVo cells.

**Table 3:** Half inhibition concentration (IC50) of candidate drugs for LoVo cells.

Drug	IC50	Drug	IC50	Drug	IC50
Apigenin	15 µM	cryptotanshinone	14 µM	curcumin	65 µM
ginsenosideRg3	30 µM	naringenin	17 µM	genistein	>100 µM
Baicalin	>100 µM	polydatin	29.5 µM	puerarin	75 µM
Luteolin	9.4 µM	echinacoside	18.6 µM	oxymatrine	>100 µM
triptolide	45 nM	resveratrol	55 µM	ursolic acid	61.5 µM
sinomenine	21.8 µM	chlorogenic acid	>100 µM	bufalin	41 nm
aloe-emodin	27 µM	osthole	43.5 µM		
hesperidin	16.4 µM	norcantharidin	16 µM		

### 3. Resveratrol Inhibits the Nuclear Localization of β-catenin, Levels of its Downstream Proteins, and MALAT1 Expression in LoVo Cells

Next, we found that resveratrol attenuated the cellular localization of β-catenin, a protein regulating cancer cell invasion and metastasis. As shown in Figure 3A, in a dose-dependent manner, resveratrol enhanced the cytoplasmic levels of β-catenin, while decreasing its presence in the nucleus, with little effect on the total cellular β-catenin protein.

**Figure 3:** Resveratrol decreases the nuclear localization of β-catenin, levels of its downstream proteins, and represses MALAT1 expression in LoVo cells. (A): Total or cell extracts of different cellular compartments from LoVo cells treated with resveratrol were probed for β-catenin. β-catenin protein levels were quantified. *p<0.05 or **p<0.01, compared with control group. (B): Total cell extracts of LoVo cells treated with resveratrol were probed for c-Myc, MMP-7 and the protein levels were quantified. *p<0.05 or **p<0.01, compared with control LoVo cells. (C): The expression levels of MALAT1 from LoVo cells treated with indicated doses of resveratrol were determined by real time PCR. The relative MALAT1 promoter activities in LoVo cells treated with indicated resveratrol doses were measured. *p<0.05 or **p<0.01, compared with control LoVo cells.

We next studied the expression of downstream β-catenin target genes in the presence of resveratrol, for the main role of β-catenin in nucleus is through its regulation on gene transcription. Unsurprisingly, we found the expression of β-catenin downstream target genes c-Myc and MMP-7 was significantly reduced by resveratrol, in a dose-dependent manner (Figure 3B). These data indicated that resveratrol may inhibit cancer cell invasion and migration through repressing Wnt/β-catenin signal pathway.

Furthermore, we discovered that resveratrol down-regulated the expression of long non-coding RNA-MALAT1 in a dose-dependent manner (Figure 3C). To verify the impact of resveratrol on MALAT1 expression, we used MALAT1 promoter dual-luciferase reporter system and found that resveratrol directly inhibited the promoter activity of MALAT1, e.g. only 10% promoter activity was achieved with 50 µM of resveratrol relative to control (Figure 3D). These data suggested that resveratrol have direct impact on the MALAT1 gene transcription.

### 4. MALAT1 Promotes the Proliferation, Invasion and Migration, and Increases the Nuclear Localization of β-catenin and Levels of its Downstream gene Products in LoVo Cells

Next, using lentivirus-mediated constructs, we knocked down or over expressed MALAT1 gene expression in LoVo cells. Our data clearly demonstrated that the proliferation and invasion/migration capability of LoVo cells were significantly decreased by MALAT1 knockdown, and increased by MALAT1 over-expression (Figure 4A, 4B).

**Figure 4:** MALAT1 promotes the proliferation, invasion and migration of LoVo cells. (A): *In vitro* growth of LoVo cells expressing MALAT1-shRNA, MALAT1-overexpression, empty vector vs. parental cells. (B): Assessment and quantification of cell migration and invasion of indicated LoVo cells in A. Values represent the number of migratory/invasive cells per 5 high power fields. *p<0.05 or **p<0.01, compared with control LoVo group.

When we knocked down, MALAT1 gene expression using shRNA construct in LoVo cells, we were surprised to find that β-catenin protein was retained in cytoplasm while its presence in nuclei was remarkedly increased (Figure 5A). Additionally, we found MALAT1 knockdown reduced the expression of β-catenin downstream target genes such as c-Myc, MMP-7, as MALAT1 over-expression did the opposite (Figure 5B). This set of data strongly implied that resveratrol inhibited the proliferation, invasion and migration properties of CRC cells via down-regulating the MALAT1 expression.

**Figure 5:** MALAT1 increases the nuclear localization of β-catenin and levels of its downstream proteins in LoVo cells. (A): Whole or cell extracts of different cellular compartments from LoVo cells expressing MALAT1-shRNA, MALAT1-overexpression, empty vector were probed for β-catenin and the protein levels were quantified. *p<0.05 or **p<0.01, compared with vector control. (B): Whole or cell extracts of different cellular compartments from LoVo cells expressing MALAT1-shRNA, MALAT1-overexpressed, empty vector were probed for c-Myc, MMP-7 and the protein levels were quantified. *p<0.05 or **p<0.01, compared with vector control.

### 5. Overexpression of MALAT1 rescues LoVo Cells from Suppressed Migration and Invasion by Resveratrol

To confirm our finding of resveratrol suppressing migration and invasion of LoVo cells through MALAT1, a MALAT1 rescue experiment was performed. Our results demonstrated that lentivirus-mediated overexpression of MALAT1 significantly attenuated resveratrol-induced inhibition on cell migration and invasion in LoVo cells (Figure 6A). In other words, overexpression of MALAT1 could reverse the effect of resveratrol. In addition, western blot results showed that overexpression of MALAT1 reversed the effect of resveratrol on nuclear β-catenin and the protein expression of c-Myc and MMP-7 in LoVo cells (Figure 6B).

**Figure 6:** Overexpression of MALAT1 attenuates the suppressive effect of resveratrol on migration and invasion in LoVo cells. (A): LoVo cells expressing MALAT1-overexpressed, empty vector were treated with or without 50 µM resveratrol for 48 hours and cellular migration and invasion ability were measured. (B): Whole or cell extracts of different cellular compartments from LoVo cells expressing MALAT1-overexpressed, empty vector treated with or without 50 µM resveratrol were probed for β-catenin, c-Myc, MMP-7, and the protein levels were quantified. *p<0.05 or **p<0.01, compared with LoVo cells treated with 50 µM resveratrol.

### 6. Resveratrol Inhibits Wnt/β-catenin Signaling via MALAT1

We hypothesized that resveratrol inhibited the Wnt/β-catenin signal pathway through MALAT1 regulation. To test this hypothesis, we used immunostaining and Western blot analyses to observe whether β-catenin trans-located from cytoplasm to nuclear with the presence of resveratrol and manipulation of MALAT1 expression levels. To make the effect more obvious, we used LiCl to inhibit the GSK3β from binding to β-catenin protein, to increase the active status of the Wnt/β-catenin signal pathway. Our results established, as LiCl indeed induced the translocation of β-catenin protein from cytoplasm to nucleus, resveratrol (50 µM) significantly impeded this process (Figure 7A). Subsequently, down-regulation of MALAT1 enhanced the effect of resveratrol on the inversion of β-catenin translocation from cytoplasm to nucleus in shRNA/MALAT1 LoVo cells, while up-regulation of MALAT1 weakened it (Figure 7B, 7C).

**Figure 7:** Resveratrol inhibits the Wnt/β-catenin signaling through regulating MALAT1. (A): Resveratrol negated LiCl induced nuclear translocation of β-catenin. Immunofluorescence staining of β-catenin in LoVo cells treated with LiCl, with or without resveratrol. (B): Nuclear extracts from LoVo cells expressing MALAT1-shRNA, MALAT1-overexpressed, empty vector, treated with LiCl with or without resveratrol, were probed for β-catenin, c-Myc, MMP-7. (C): Quantification of β-catenin, c-Myc, MMP-7 protein levels from the data shown in (A). **p<0.01, compared with blank group or LiCl alone group. (D): The relative LEF/TCF promoter activities in LoVo cells expressing MALAT1-shRNA, MALAT1-overexpressed, empty vector, treated by LiCl, with or without resveratrol. **p<0.01, compared with blank group or LiCl alone group. (E): No interaction between MALAT1 and β-catenin. Insert: RT-PCR result showing amount of RNA pulled-down by RNA-binding protein immunoprecipitation. As negative controls, no cDNA (blank) or IgG alone was used. Lower pane: quantification result of the insert.

Moreover, we tested the effect of resveratrol on Wnt/β-catenin signaling using a reporter LEF/TCF promoter dual-luciferase construct. Our results clearly indicated that, resveratrol inhibited the promoter activity of LEF/TCF induced by LiCl, and co-repression of MALAT1 led to the enhancement of this effect, as co-overexpression of MALAT1 opposing it (Figure 7D). All these data underpinned that resveratrol inhibits the activity of Wnt/β-catenin signal pathway via repressing the MALAT1 expression. Since MALAT1 and β-catenin protein both exist in the nucleus, so it is of great interest for us to know whether these two molecules can directly interact with each other, which can be detected using a RNA-binding protein immunoprecipitation technique. Surprisingly, our data showed little interaction between MALAT1 and β-catenin (Figure 7E). This illustrated that MALAT1 might indirectly interact with β-catenin to affect its signal cascade.

### 7. Corroboration of our Key Findings in Another CRC Cell Line HCT116

To confirm our key findings in LoVo cells, we tested another CRC HCT116 cell line using similar approaches. Our results showed that resveratrol inhibited the proliferation of HCT116 cells by the IC50 of 100 µM (Figure 8A). HCT 116 cells had much lower MALAT1 expression than LoVo cells, but nonetheless, as similar to LoVo cells, overexpression of MALAT1 promoted the proliferation of HCT116 cells (Figure 8B, 8C, 8D).

**Figure 8:** Resveratrol inhibits the Wnt/β-catenin signaling through regulating MALAT1.in CRC HCT116 cells. (A): Resveratrol inhibited the proliferation of HCT116 cells with an IC50 of 100 µM. (B): HCT 116 cells showed lower MALAT1 expression than LoVo cells. **p<0.01, compared with LoVo cells. (C): Overexpression of MALAT1 in HCT116 cells. (D): Overexpression of MALAT1 promoted the in vitro growth of HCT116 cells. (E): Overexpression of MALAT1 attenuated the suppressive effect of resveratrol on migration and invasion in HCT116 cells. HCT116 cells expressing MALAT1-overexpressed, empty vector were treated with or without 50 µM resveratrol for 48 hours and cellular migration and invasion ability were measured. (F): Whole or cell extracts of different cellular compartments from HCT116 cells expressing MALAT1-overexpressed, empty vector treated with or without 50 µM resveratrol for 48 hours were probed for β-catenin, c-Myc, MMP-7 and the protein levels were quantified. *p<0.05 or **p<0.01, compared with HCT116 cells treated with 100 µM resveratrol.

In addition, resveratrol also significantly inhibited the migration and invasion ability of HCT116. As in LoVo cells, overexpression of MALAT1 rescued HCT116 cells from suppression of migration and invasion by resveratrol (Figure 8E). Western blot results also showed that overexpression of MALAT1 reversed the effect of resveratrol on nuclear β-catenin and the protein expression of c-Myc and MMP-7 in HCT116 cells (Figure 8F).

## Discussion

Colorectal cancer is one of the most common malignant tumors in the world, with high rate of recurrence and metastasis. The mechanisms of recurrence and metastasis remain very complicated. Currently, the treatment of colorectal cancer is mainly surgical resection, combined with chemotherapy, immunotherapy, and other alternative cares such as traditional Chinese medicine. Traditional Chinese medicine and its more recently derived extracted monomer treatment can improve cancer symptoms, reduce cancer metastasis, as well as reduce the risk of recurrence of colorectal cancer. However, the therapeutic targets and mechanisms remain elusive. Among these extracted monomers, resveratrol is a perfect example. As early as in 1993, Jayafilake *et al* has found that resveratrol has anti-cancer characteristic because of its repressive effect on protein-tyrosine kinase activity [20]. Other researchers further found that resveratrol has inhibitory effect on a great spectrum of malignant tumor cells derived from breast, gastric, colon, prostate, ovarian, and skin cancers [21]–[26]. Our current studies demonstrated that resveratrol inhibits the proliferation, invasion and metastasis of colorectal cancer cells.

Being the key transcriptional activation factor of Wnt/β-catenin signal pathway, upon upstream activation, β-catenin often translocates to the nucleus from cytoplasm, in coordination with other transcription factors such as TCF/LEF, to activate its target genes c-Myc, cyclinD1, MMP-7, and CD44, which in turn play pivotal role in tumor initiation and development [27]–[30]. Our data indicated that resveratrol blocked the translocation of β-catenin to nucleus, resulting in lowered expression of c-Myc and MMP-7.

Long non-coding RNA-MALAT1 was firstly reported in the invasive non-small cell carcinoma, and lately being found over-expressing in many other cancer tissues, that indicated MALAT1 is associated with invasion and metastasis [11]–[14]. Our studies showed MALAT1 over-expressed in 60 CRC tissues compared to the adjacent normal tissues, and MALAT1 overexpression correlated with CRC invasion and metastasis features. In our screening experiments, we have identified two traditional Chinese medicine extracted monomers which have direct effect on MALAT1 expression. Resveratrol is the best of them. In our current studies, we illustrated that shRNA mediated knockdown of MALAT1 obviously reduced invasion and migration capabilities of CRC LoVo and HCT116 cells. Similar to the results of resveratrol treatment, knockdown of MALAT1 inhibited the trans-location of β-catenin from cytoplasm to nucleus, resulting in decreased c-Myc and MMP-7 expression, while MALAT1 over-expression did the opposite.

By using a LEF/TCF promoter dual-luciferase reporter construct and activating the Wnt/β-catenin signal pathway with LiCl, we further demonstrated that knockdown of MALAT1 enhanced the inhibitory effect of resveratrol on the promoter activity of LEF/TCF induced by LiCl, while over-expression of MALAT1 weakened it. All these results suggested that the underlining mechanism of resveratrol may be through a repression of Wnt/β-catenin signaling, via down-regulation of MALAT1 expression.

MALAT1 is specifically retained in nuclear speckles, associated with storage or modification of the pre-mRNA processing machinery, has potential effect on gene function regulation, all these imply that MALAT1 can play an important role in carcinogenesis [31]–[33]. For the reason that MALAT1 and β-catenin protein both reside in the nucleus, we examined whether there is a direct interaction between these two molecules in the nucleus. Unfortunately we observed little direct interaction between MALAT1 and β-catenin, suggesting that there might be other molecules involved in the regulation between MALAT1 and β-catenin. No direct correlation between high MALAT1 expression in clinical samples and nuclear accumulation of β-catenin was found. As proposed by Brabletz T *et al*, β-catenin (Figure S1) in colon carcinomas showed a strong nuclear enrichment at the invasion front, whereas in large parts of the central tumor area, β-catenin was detected in the cytoplasm and at the membrane [34]–[36]. This means that we should separate the invasion front from the rest of the CRC tissue and measure expression levels of MALAT1, β-catenin and their localization, for their correlation. We plan in future studies, using technologies such as prediction analysis software, co-immunoprecipitation, protein sequencing, protein chips and gene chips, to identify the specific links between MALAT1 and β-catenin.

In conclusion, our results uncovered the mechanisms by which resveratrol regulates MALAT1, in turn alters the nuclear localization of β-catenin, resulting in lowered Wnt/β-catenin signaling and eventual inhibition of invasion and metastasis. This discovery will surely provide vital pre-clinical evidence supporting future use of resveratrol in prevention and treatment of CRC.

## Supporting Information

Figure S1 **Selection of the most efficient shRNA for MALAT1, detection of MALAT1 mRNA and β-catenin protein expression in CRC tissues and adjacent normal tissues.** (A): LoVo cells were infected with the lentivirus with three pLV4-MALAT1 shRNAs or pLV4-vector. Their efficiencies of knockdown were detected by real time PCR.*p<0.05 or **p<0.01, compared with vector control. (B): MALAT1 mRNA expression levels were measured by real time PCR, CRC tissues and adjacent normal tissues. **p<0.01, compared with normal tissues or CRC tissues with no metastasis. (C): Immunofluorescent staining of β-catenin in CRC tissues and adjacent normal tissues.
(TIF)

## References

[1] FidlerIJ (2003) The pathogenesis of cancer metastasis: the seed and soil hypothesis revisited. Nat Rev Cancer 3: 1–6.10.1038/nrc109812778135

[2] XuTM, CuiMH, XinY, GuLP, JiangX, et al (2008) Inhibitory effect of ginsenoside Rg3 on ovarian cancer metastasis. Chin Med J 121: 1394–1397.18959116

[3] ChangJS, LiuHW, WangKC, ChenMC, ChiangLC, et al (2005) Ethanol extract of Polygonum cuspidatum inhibits hepatitis B virus in a stable HBV-producing cell line. Antiviral Res 66: 29–34.1578112910.1016/j.antiviral.2004.12.006

[4] ChinYH, YuPC, JeliC (2007) Antioxidant activity of extract from Polygonum cuspidatum. Biol Res 40: 13–21.1765735110.4067/s0716-97602007000100002

[5] FengL, ZhangLF, YanT, JinJ, TaoWY (2006) Studies on active substance of anticancer effect in Polygonum cuspidatum. Zhong Yao Cai 29: 689–691.17059010

[6] ShinJA, ShimJH, JeonJG, ChoiKH, ChoiES, et al (2011) Apoptotic effect of Polygonum Cuspidatum in oral cancer cells through the regulation of specificity protein 1. Oral Dis 17: 162–170.2065926410.1111/j.1601-0825.2010.01710.x

[7] WuXB, LuoXQ, GuSY, XuJH (2012) The effects of Polygonum cuspidatum extract on wound healing in rats. J Ethnopharmacol 141: 934–937.2246976810.1016/j.jep.2012.03.040

[8] De la LastraCA, VillegasI (2007) Resveratrol as an antioxidant and pro-oxidant agent: mechanisms and clinical implications. Biochem Soc Trans 35: 1156–1160.1795630010.1042/BST0351156

[9] OlasB, WachowiczB (2005) Resveratrol, a phenolic antioxidant with effects on blood platelet functions. Platelets 16: 251–260.1601197510.1080/09537100400020591

[10] AtharM, BackJH, TangX, KimKH, KopelovichL, et al (2007) Resveratrol: a review of preclinical studies for human cancer prevention. Toxicol Appl Pharm 224: 274–283.10.1016/j.taap.2006.12.025PMC208312317306316

[11] JiP, DiederichsS, WangW, BoingS, MetzgerR, et al (2003) MALAT-1, a novel noncoding RNA, and thymosin b4 predict metastasis and survival in early-stage non-small cell lung cancer. Oncogene 22: 8031–8041.1297075110.1038/sj.onc.1206928

[12] LinR, MaedaS, LiuC, KarinM, EdgingtonTS (2007) A large noncoding RNA is a marker for murine hepatocellular carcinomas and a spectrum of human carcinomas. Oncogene 26: 851–858.1687814810.1038/sj.onc.1209846

[13] GuoFJ, LiYL, LiuY, WangJJ, LiYH, et al (2010) Inhibition of metastasis-associated lung adenocarcinoma transcript 1 in CaSki human cervical cancer cells suppresses cell proliferation and invasion. Acta Biochim Biophys Sin 42: 224–229.2021304810.1093/abbs/gmq008

[14] XuC, YangM, TianJ, WangX, LiZ (2011) MALAT-1: a long non-coding RNA and its important 3’ end functional motif in colorectal cancer metastasis. Int J Oncol 39: 169–175.2150357210.3892/ijo.2011.1007

[15] IwaiS, YonekawaA, HaradaC, HamadaM, KatagiriW, et al (2010) Involvement of the Wnt-β-catenin pathway in invasion and migration of oral squamous carcinoma cells. Int J Oncol 37: 1095–1103.2087805710.3892/ijo_00000761

[16] GuoQ, ShenS, LiaoM, LianP, WangX (2010) NGX6 inhibits cell invasion and adhesion through suppression of Wnt/β-catenin signal pathway in colon cancer. Acta Biochim Biophys Sin 42: 450–456.2070558310.1093/abbs/gmq049PMC2948811

[17] TannerM, GancbergD, LeoAD, LarsimontD, RouasG, et al (2000) Chromogenic *in situ* hybridization: a practical alternative for fluorescence *in situ* hybridization to detect HER-2/neu oncogene amplification in archival breast cancer samples. Am J Pathol 157: 1467–1472.1107380710.1016/S0002-9440(10)64785-2PMC1885742

[18] FungH, DempleB (2005) A vital role for Ape1/Ref1 protein in repairing spontaneous DNA damage in human cells. Mol Cell 17: 463–470.1569434610.1016/j.molcel.2004.12.029

[19] KweiderN, FragoulisA, RosenC, PecksU, RathW, et al (2011) Interplay between vascular endothelial growth factor (VEGF) and nuclear factor erythroid 2-related factor-2 (Nrf2): implications for preeclampsia. J Biol Chem 286: 42863–42872.2203392310.1074/jbc.M111.286880PMC3234879

[20] JayatilakeGS, JayasuriyaH, LeeES, KoonchanokNM, GeahlenRL, et al (1993) Kinase inhibitors from Polygonum cuspidatum. J Nat Prod 56: 1805–1810.827731810.1021/np50100a021

[21] GarvinS, ÖllingerK, DabrosinC (2006) Resveratrol induces apoptosis and inhibits angiogenesis in human breast cancer xenografts *in vivo* . Cancer Lett 231: 113–122.1635683610.1016/j.canlet.2005.01.031

[22] RilesWL, EricksonJ, NayyarS, AttenMJ, AttarBM, et al (2006) Resveratrol engages selective apoptotic signals in gastric adenocarcinoma cells. World J Gastroenterol 12: 5628–5634.1700701410.3748/wjg.v12.i35.5628PMC4088162

[23] PanaroMA, CarofiglioV, AcquafreddaA, CavalloP, CianciulliA (2012) Anti-inflammatory effects of resveratrol occur via inhibition of lipopolysaccharide-induced NF-κB activation in Caco-2 and SW480 human colon cancer cells. Br J Nutr 108: 1623–1632.2225162010.1017/S0007114511007227

[24] HudsonTS, HartleDK, HurstingSD, NunezNP, WangTT, et al (2007) Inhibition of prostate cancer growth by muscadine grape skin extract and resveratrol through distinct mechanisms. Cancer Res 67: 8396–8405.1780475610.1158/0008-5472.CAN-06-4069

[25] NessaMU, BealeP, ChanC, YuJQ, HuqF (2012) Combinations of resveratrol, Cisplatin and oxaliplatin applied to human ovarian cancer cells. Anticancer Res 32: 53–59.22213288

[26] BackJH, ZhuY, CalabroA, QueenanC, KimAS, et al (2012) Resveratrol-mediated downregulation of rictor attenuates autophagic process and suppresses UV-induced skin carcinogenesis. Photochem Photobiol 88: 1165–1172.2227277510.1111/j.1751-1097.2012.01097.xPMC7703848

[27] LiZR, WuYF, MaCY, NieSD, MaoXH, et al (2011) Down-regulation of c-Myc expression inhibits the invasion of bile duct carcinoma cells. Cell Biol Int 35: 799–802.2155772610.1042/CBI20110099

[28] ZhangJ, GillAJ, IssacsJD, AtmoreB, JohnsA, et al (2012) The Wnt/β-catenin pathway drives increased cyclin D1 levels in lymph node metastasis in papillary thyroid cancer. Hum Pathol 43: 1044–1050.2220471310.1016/j.humpath.2011.08.013

[29] VillarJ, CabreraNE, ValladaresF, CasulaM, FloresC, et al (2011) Activation of the Wnt/β-Catenin signaling pathway by mechanical ventilation is associated with ventilator-induced pulmonary fibrosis in healthy lungs. PLoS ONE 6: e23914.2193536510.1371/journal.pone.0023914PMC3174135

[30] ZeilstraJ, JoostenSP, DokterM, VerwielE, SpaargarenM, et al (2008) Deletion of the WNT target and cancer stem cell marker CD44 in Apc(Min/+) mice attenuates intestinal tumorigenesis. Cancer Res 68: 3655–3661.1848324710.1158/0008-5472.CAN-07-2940

[31] HutchinsonJN, EnsmingerAW, ClemsonCM, LynchCR, LawrenceJB, et al (2007) A screen for nuclear transcripts identifies two linked noncoding RNAs associated with SC35 splicing domains. BMC Genomics 8: 39.1727004810.1186/1471-2164-8-39PMC1800850

[32] WiluszJE, FreierSM, SpectorDL (2008) 3′-end processing of a long nuclear retained noncoding RNA yields a tRNA-like cytoplasmic RNA. Cell 135: 919–932.1904175410.1016/j.cell.2008.10.012PMC2722846

[33] LaiMC, YangZ, ZhouL, ZhuQQ, XieHY, et al (2012) Long non-coding RNA MALAT-1 overexpression predicts tumor recurrence of hepatocellular carcinoma after liver transplantation. Med Oncol 29: 1810–1816.2167802710.1007/s12032-011-0004-z

[34] BrabletzT, JungA, ReuS, PorznerM, HlubekF, et al (2001) Variable beta-catenin expression in colorectal cancers indicates tumor progression driven by the tumor environment. Proc Natl Acad Sci USA 98: 10356–10361.1152624110.1073/pnas.171610498PMC56965

[35] BrabletzT, JungA, DagS, ReuS, KirchnerT (2000) beta-Catenin induces invasive growth by activating matrix metalloproteinases in colorectal carcinoma. Verh Dtsch Ges Pathol 84: 175–181.11217438

[36] HlubekF, BrabletzT, BudcziesJ, PfeifferS, JungA, et al (2007) Heterogeneous expression of Wnt/beta-catenin target genes within colorectal cancer. Int J Cancer 121: 1941–1948.1763164110.1002/ijc.22916

